# Optimization of Tumor Disease Monitoring in Medical Big Data Environment Based on High-Order Simulated Annealing Neural Network Algorithm

This article has been retracted.

**DOI:** 10.1155/2021/8996673

**Published:** 2021-10-19

**Authors:** Lei Zhang, Qixiang Zhong, Zhenglun Yu

**Affiliations:** ^1^Department of Breast Surgery, The First Affiliated Hospital of China Medical University, Shenyang, Liaoning 110001, China; ^2^Department of Thoracic Surgery, The First Affiliated Hospital of China Medical University, Shenyang, Liaoning 110001, China

## Abstract

With the development of medical informatization, the data related to medical field are growing at an amazing speed, and medical big data appears. The mining and analysis of these data plays an important role in the prediction, monitoring, diagnosis, and treatment of tumor diseases. Therefore, this paper proposes a clustering algorithm of the high-order simulated annealing neural network algorithm and uses this algorithm to extract tumor disease-related big data, constructs training set according to the relevant information mined, designs a kind of dimension reduction model, aiming at the problem of excessive and wrong diagnosis and treatment in the diagnosis and treatment module of tumor disease monitoring mode, and establishes the corresponding control mechanism, so as to optimize the tumor disease monitoring mode. The results show that the clustering accuracy of the high-order simulated annealing neural network algorithm on different data sets (iris, wine, and Pima India diabetes) is 97.33%, 82.11%, and 70.56% and the execution time is 0.75 s, 0.562 s, and 1.092 s, which are better than those of the fast *k*-medoids algorithm and improved *k*-medoids clustering algorithm. To sum up, the high-order simulated annealing neural network algorithm can achieve good clustering effect in medical big data mining. The establishment of model M1 can reduce the probability of excessive and wrong medical treatment and improve the effectiveness of diagnosis and treatment module monitoring in tumor disease monitoring mode.

## 1. Introduction

With the rapid development of medical informatization, medical data are growing rapidly, and the era of medical big data is coming. In the field of diagnosis and treatment of malignant tumor, the diagnosis, prevention, and monitoring of malignant tumor all run through the collection, management, and corresponding analysis of data [1]. Cancer disease monitoring mode is an effective measure to increase the prevention and treatment of cancer. The tumor disease monitoring mode is based on the mining and monitoring of partial and all information of different stages, such as pretumor, tumorigenesis, and tumor development [2]. At present, there is no perfect tumor disease monitoring mode, and there is no complete monitoring system for tumor information [3]. Tumor-related information in the tumor information monitoring system is mainly provided by chronic disease and nutrition monitoring system, cause of death monitoring system, and tumor registration system. These three information systems are also important references for establishing the tumor disease information system [4]. The chronic disease and nutrition monitoring system is mainly responsible for monitoring the patients with chronic diseases and related factors, the trend of nutritional diseases, and so on. The cause of death detection system is mainly responsible for studying the death level of population and plays an important role in optimizing the allocation of resources and evaluating the health of residents; the cancer registration system is mainly responsible for collecting cancer incidence and survival status information of residents so as to show the epidemic trend of cancer. Therefore, it is particularly important to study medical big data tumor disease monitoring methods, which has become a research hotspot in the current medical field.

Mundada et al. designed a processing optimization scheme combining the simulated annealing algorithm and artificial neural network algorithm, which can significantly improve the productivity [5]. Zhang et al. proposed to use the simulated annealing genetic algorithm to optimize the back-propagation process of neural network to simulate the fault diagnosis of autopilot flight control box [6]. Hua et al. put forward a fault diagnosis strategy of chiller based on deep neural network and simulated annealing genetic algorithm [7]. Khan and Shaikh built a functional connection between simulated annealing neural network and Legendre polynomial artificial neural network and verified the effectiveness of the link by controlling the nonlinear Lane Emden singular initial value problem of multidirectional and isothermal gas sphere [8]. Ji et al. proposed to find the optimal solution through the combination of the simulated annealing algorithm and Nder-Mead simplex algorithm [9]. Aiming at the current situation that the accuracy of flatness prediction methods cannot meet the standard, scholars Xiu et al. proposed a flatness prediction model based on digital signal processor combined with T-S cloud reasoning network. The model effectively combines the simulated annealing algorithm and genetic algorithm. The experimental results show that the prediction model has ideal robustness and accuracy [10].

Dlamini et al. discussed that artificial intelligence (AI) has significantly influenced many facets of the healthcare sector. Through these applications of AI, cancer diagnostics and prognostic prediction are enhanced with medical imaging that delivers high resolution images [11]. Abd El Kader et al. proposed a differential deep convolutional neural network model (differential deep-CNN) to classify different types of brain tumor, including abnormal and normal magnetic resonance (MR) images [12]. Woźniak et al. proposed a novel correlation learning mechanism (CLM) for deep neural network architectures that combines convolutional neural network (CNN) with classic architecture to detect brain tumor [13]. Wang et al. has proposed a learning scheme of nuclear extreme learning machine (KELM) based on chaos moth flame optimization (CMFO) strategy. Using Parkinson's disease and breast cancer's medical diagnosis problem, the proposed method is compared with other competing KELM models based on original moth flame optimization, particle swarm optimization, and genetic algorithm. Experimental results show that compared with other methods, this method has better classification performance and obtains smaller feature subsets. [14]. Luo et al. explored the value of liquid biopsy technology in tumor diagnosis, prognosis prediction, and disease monitoring. This study shows that liquid biopsy has strong feasibility and can bring good news to many subsequent cancer patients [15].

To sum up, the current research on medical big data tumor disease monitoring mode is mostly the optimization and improvement of medical technology, while the research on medical big data tumor disease monitoring mode is relatively less and has not achieved ideal results. At the same time, the high-order simulated annealing neural network algorithm has been widely used in all walks of life and achieved satisfactory results. Because the medical data are usually large, we can further mine the medical big data through the K-medoid algorithm of data mining. In view of this, this study proposes to optimize the medical big data tumor disease monitoring mode by using the high-order simulated annealing neural network algorithm, aiming to provide scientific guidance for the intervention treatment of cancer patients.

## 2. Optimization of Neural Network Algorithm Based on High-Order Simulated Annealing

### 2.1. Research on Medical Big Data Mining Technology Based on High-Order Simulated Annealing Neural Network Algorithm

Firstly, it is clear that medical big data is a kind of big data, which has 4 V characteristics such as large volume, real-time, diversity, and uncertainty [16–22]. Therefore, the research combines the *K*-medoid algorithm with the high-order simulated annealing neural network algorithm to mine medical big data. Due to the deficiency of random selection of initial center point in the *K*-medoid algorithm, this paper studies the effective initialization of the *K*-medoid algorithm through improved granular computing [23]. Suppose that *T*=(*X*, *B*) is the clustering space, the sample object set is *U*, and the attribute set is *B*, then the sample object similarity *S*(*x*_*i*_, *x*_*j*_) satisfies the following conditions:

(1) $$\begin{array}{c} S\left(x_{i},x_{j}\right)=\frac{1}{\left(1+\sum_{l=1}^{\left|B\right|}w_{l}\left|x_{il}-x_{jl}\right|\right)}. \end{array}$$

In formula (1), *W*_*l*_ is the attribute resolution and is used to describe the proportion of attribute value in the corresponding object set; *l* represents attribute value, which is divided into interval block {*x*_1_, *x*_2_,…, *x*_*m*_}; *m* is the number of partition blocks; and both *x*_*i*_ and *x*_*j*_ represent sample objects.

(2) $$\begin{array}{c} w_{l}=\frac{\sum_{i=1}^{m}{\left|x_{i}\right|}^{2}}{{\left|U\right|}^{2}}, \end{array}$$

where |*x*_*i*_| is the number of objects in the partition interval of *x*_*i*_; *m* is the number of partition blocks; and |*U*| represents the total number of objects. When the number of sample objects is *n*, the average similarity of sample objects $\bar{d}$ can be obtained as follows:

(3) $$\begin{array}{c} \bar{d}=\frac{\sum_{i,j=1}^{n}S\left(x_{i},x_{j}\right)}{n^{2}}, \end{array}$$

where *S*(*x*_*i*_, *x*_*j*_) represents the similarity of sample objects and *n* is the number of sample objects.

(4) $$\begin{array}{c} gd\left(X_{i}\right)=\frac{\left|x_{i}\right|}{\left|U\right|}. \end{array}$$

Formula (4) is the formula for calculating the density *gd*(*X*_*i*_) of particle *X*_*i*_, where *U* represents the object set, and the particles with *n* on the object set are divided into {*X*_1_, *X*_2_,…, *X*_*n*_}; *n* is the number of sample objects; |*X*_*i*_| is the number of sample objects in the *i*-th interval.

(5) $$\begin{array}{c} \bar{GD}=\frac{\sum_{i=1}^{n}gd\left(X_{i}\right)}{n}. \end{array}$$

Equation (5) is the average density of particles $\bar{GD}$'s calculational formula, where *n* represents the number of particles in a set of objects *U*. When the *i*-th particle has *N* objects, they are *x*_*i*1_, *x*_*i*2_,…, *x*_*iN*_. The definition formula of the center of the particle *O*_*i*_ is as follows:

(6) $$\begin{array}{c} o_{i}=\left\{x_{ij}|\overset{N}{\underset{j=1}{\min}}\left|x_{ij}-\frac{1}{N}\overset{N}{\underset{k=1}{\sum }}x_{ik}\right|\right\}. \end{array}$$

In equation (6), *N* refers to the *N* objects existing in the *i*th particle. Set the threshold *d*, when *S*(*x*_*i*_, *x*_*j*_) ≥ *d*, *M*(*i*, *j*)=1. When *S*(*x*_*i*_, *x*_*j*_) < *d*, then *M*(*i*, *j*)=0, where *M* is the adjacency similarity matrix between sample objects. The rough set *G* is obtained by classifying the object matrix *M*. After reprocessing, the number of samples is arranged in order of size, and the samples *G* are not repeated. The average density of fine particle set *G* is calculated by equation (5), and the particles of *gd*(*x*_*i*_) ≥ *GD* are regarded as effective particles and put into effective particle set *I*. The Euclidean distance between any two particles and the centers of different particles in the effective particle set *I* are obtained by equation (6), and the Euclidean distance is recorded in the set *D*. In *I*, the center with the largest particle density is selected as the first center point *O*_1_, and the corresponding particle is labeled as *Q*_1_. The center point corresponding to the particle which is the farthest from the particle with the largest density at the same time acts as the second center point *O*_2_, and the particles corresponding to each other are labeled as *Q*_2_. According to *D*, the distance between the remaining particles in the set *I* and the center point *O*_1_, *O*_2_,…, *O*_*n*_ is calculated in turn, that is, *d*_*i*1_, *d*_*i*2_,…, *d*_*in*_. At the same time, we make *d*_*i*_=min(*d*_*i*1_, *d*_*i*2_,…, *d*_*in*_) and then calculate max(*d*_*i*_). At the same time, we mark the center point of the corresponding particles as *O*_*i*_ and the particles as *Q*_*i*_ and so on to *O*_*k*_ and *Q*_*k*_ [19, 20]. Then, the *K*-medoid algorithm is initialized effectively. The annealing simulation algorithm has the characteristics of high efficiency, robustness, versatility, and flexibility [21] In equation (6), *N* refers to the second *i*. Set threshold *d*, when *S*(*x*_*i*_, *x*_*j*_) ≥ *d*, then *M* (*i*, *j*) = 1; when *S*(*x*_*i*_, *x*_*j*_) < *d*, then *M* (*i*, *j*) = 0 of which *M* is the adjacency similarity matrix between sample objects. By analyzing the object matrix*M*, the rough set can be obtained by classifying *G*. After reprocessing, the number of samples is arranged in the order of size, and the samples are not repeated *G*; the fine-grained set is calculated by equation (5) *G*. The ratio of the two average densities can be obtained *gd*(*x*_*i*_) ≥ *GD*. As effective particles, put them into effective particle set *I* medium. The effective particle set is obtained by equation (6) *I*. The Euclidean distance between any two particles is recorded in the set *D* in the middle. *I* select the center with the highest particle density as the first center point *O*_1_, the corresponding particle is marked as *O*_1_. The center point corresponding to the particle with the farthest distance from the maximum density particle and the maximum density of itself is taken as the second center point *O*_2_. The particles corresponding to each other are labeled as *O*_2_; According to *D*, find the distance from the remaining particles in the model to the central points *O*_1_, *O*_2_, *O*_3_, in turn. This distance is marked as set *I*. Mark the corresponding particle center as *O*_*i*_, particles labeled as *O*_*i*_, and so on *O*_*k*_, *O*_*k*_ [24, 25]. Then, the *K*-medoid algorithm is initialized effectively. The annealing simulation algorithm has the characteristics of high efficiency, robustness, versatility, and flexibility [26].

The criterion function of the traditional *k*-medoids clustering algorithm is shown in formula (1), and the distance and minimum within the cluster are considered as the criteria to measure the clustering quality. The core idea of clustering is to require the minimum distance within clusters and the maximum distance between clusters. Equation (1) only considers the distance within clusters and ignores that the overall quality of clustering is determined by the distance within clusters and the distance between clusters. Based on the above ideas, a class of criterion functions for balancing the distance within and between clusters is given, as shown in equation (7). If the new criterion function reaches the minimum value, the optimal clustering result can be obtained. Let the distance *O*(*w*) between clusters be the distance between the center points of each cluster, as shown in the following equation:

(7) $$\begin{array}{c} O\left(w\right)=\sum_{i,j=1}^{k}\left|o_{i}-o_{j}\right|. \end{array}$$

The improved criterion function can be expressed as the following equation:

(8) $$\begin{array}{c} F\left(w\right)=\frac{\sqrt{O\left(w\right)}}{\sqrt{E}}. \end{array}$$

Figure 1 shows that after setting the initial solution in the simulated annealing algorithm, including the initial temperature, the end temperature, and the annealing rate, the objective function value is calculated, and the random disturbance of the current solution is carried out according to a specific value, and then the function value of the new solution is calculated; according to the Metropolis criterion, the new solution is accepted or not. When the new solution is accepted, the old solution is replaced by the new one to cool down. When the new solution is not accepted, keep the old solution unchanged and cool down. when the current temperature is lower than the end temperature, end the algorithm and get the final solution [27, 28].

The clustering process of the hybrid network algorithm of the *K*-medoid algorithm and high-order annealing neural network algorithm:

 
*Input*. Data set *D* including *n* sample objects, number of clusters *K*.
 
*Output*. The center point of *K* clusters and the set of optimal clusters.
Step 1. The initial cluster center *o*_1_, *o*_2_,…, *o*_*n*_ is generated according to the granular calculation, which is recorded as *w*_0_. Then, the criterion function *F* (*w*_0_) is calculated, the initialization temperature is *t*_*s*_, the termination temperature is *t*_*e*_, and the maximum number of inner layer cycles at each temperature *T* is loop.
Step 2. The random disturbance generates a new center point *o*_1_′, *o*_2_′,…, *o*_*n*_′, which is recorded as *w*′, the value *F* (*w*′) of the criterion function is calculated, and then the value-added △*F* = *f* (*w*′) − *f* (*w*) of the function is calculated.
Step 3. According to the Metropolis criterion and in combination with the criterion function, if △*f* ≥ 0, the new interpretation is taken as the current interpretation; otherwise, the new solution is received with probability *P*. If a new solution is received, change *w*′ to *w* where *P*=*e*^−[*F*(*w*′) − *f*(*w*)/*Ht*]^, in which *t* is the current temperature.
Step 4. For inner layer circulation, turn to step 2 until the number of inner layer circulation finally reaches loop and turn to step 5.
Step 5. The temperature of *T* is decreased, that is, *t* (*k*) = at (*k* − 1), *k* are the times of cooling, and then turn to step 2 to step 4. Until the termination condition is satisfied: *t* (*k*) is less than *t*_*c*_, the output result and the end algorithm are finished.

In the process of calculating criterion function $F\left(w\right)=\sqrt{O\left(w\right)}/\sqrt{E}$, *O*(*w*) is the distance between the center of each cocoon and *E* is the total cost of exchanging the noncluster center object with the center object.

### 2.2. Optimization of Medical Big Data Tumor Disease Monitoring Mode

In this study, the tumor disease monitoring mode is summarized as risk factor monitoring, early detection and screening factor monitoring, tumor diagnosis and treatment factor monitoring, and tumor prognosis factor monitoring [29]. See Figure 2 for details.

As shown in Figure 2, in the risk factor monitoring under the tumor disease monitoring mode, it mainly carries out the monitoring of personal factors, environmental factors, behavior mode, and genetic factors of tumor patients; in the early detection and screening monitoring of tumor diseases, it mainly includes the monitoring of early symptoms and screening information. In tumor disease diagnosis and treatment monitoring and tumor prognosis monitoring, we mainly monitor tumor diagnosis information, tumor treatment information, and tumor prognosis information. However, with the emergence of a variety of tumor treatment drugs and treatment methods, there are errors and excessive medical problems in the treatment of tumor diseases, and the above tumor disease monitoring mode cannot effectively monitor and guide it [30]. In order to solve this problem, a medical detection and control mechanism for cancer diseases is established, and the introduction of this mechanism is used to optimize the cancer disease monitoring mode.

Firstly, the classification model of over treatment and wrong treatment is established, and the benign and malignant samples corresponding to a certain tumor disease are used as the overall training sample set *D*={(*x*_1_, *y*_1_), (*x*_2_, *y*_2_),…, (*x*_*m*_, *y*_*m*_)}, of which *x*_*i*_ is extracted through the image data extraction in pathology, which belongs to the characteristic parameters of different images, and *y*_*i*_ is the true benign and malignant grade of the tumor:

(9) $$\begin{array}{c} \omega^{T}x+b=0. \end{array}$$

Equation (9) is the expression of dividing hyperplane; normal vector *w*=(*w*_1_, *w*_2_, *w*_3_,…, *w*_*d*_) is to determine the direction of the hyperplane; displacement term *b* mainly determines the distance between the hyperplane and the origin. It can be seen that the partition hyperplane can be determined by *w* and *b*, denoted as (*w*, *b*):

(10) $$\begin{array}{c} \gamma =\frac{\left|\omega^{T}x+b\right|}{\left\|\omega \right\|}. \end{array}$$

Equation (10) is the calculation formula of distance *r* from any point in the sample space to the hyperplane (*w*, *b*). When the hyperplane (*w*, *b*) can correctly classify the training samples *y*_0_ and *y*_1_, there is (*x*_*i*_, *y*_*i*_) ∈ *D*:

(11) $$\begin{array}{c} \left\{\begin{array}{cc} \omega^{T}x+b\geq +1, & y_{i}=y_{1},\\ \omega^{T}x+b\leq -1, & y_{i}=y_{0}. \end{array}\right. \end{array}$$

As shown in equation (11), when *y*_*i*_ belongs to the classification target disease *y*_1_, there is *w*^*T*^*x*+*b* > 0. When *y*_*i*_ does not belong to the classification target disease, there is *w*^*T*^*x*+*b* < 0. The training sample points that can make equation (11) tenable can be regarded as the corresponding medical record image data (support vector); at this time, the sum of the distance between the two heterogeneous support vectors and the hyperplane *γ* is *r*:

(12) $$\begin{array}{c} \gamma =\frac{2}{\left\|\omega \right\|}. \end{array}$$

The sum of the distance between the two heterogeneous support vectors obtained by equation (12) is called “interval.” Because there are many clinical features of some tumor diseases, the data dimension of training samples is more than a certain range, which leads to the problem of over fitting, so it is necessary to implement feature selection for training data. Recursive feature elimination (RFE) algorithm + support vector machine (SVM), namely, SVM_RFE feature selection algorithm is a feature sorting and selection algorithm based on support vector machine. The implementation steps of the algorithm are shown in equations (13)–(15).

(13) $$\begin{array}{c} \alpha =\text{SVM}-\text{train}\left(X,y\right), \end{array}$$

where (13) *α* is the classifier parameter, *X* is the type of tumor, *y* represents the characteristic property of tumor, and SVM refers to the daily operator vector of support vector machine.

(14) $$\begin{array}{c} \omega =\sum_{k}\alpha_{k}y_{k}X_{k}, \end{array}$$

where (14) *w* represents the weight vector of any eigenvector *k* in the input space, *α* is the classifier parameter, *X* is the type of tumor, and *y* represents the characteristic property of tumor.

(15) $$\begin{array}{c} R_{c}=\left|\omega^{2}-\omega^{-{\left(p\right)}^{2}}\right|. \end{array}$$

In equation (15), *R*_*c*_ refers to the overall weight and puts forward the *p* th absolute value of support vector machine weight difference after feature selection. Among them, *w*^2^ refers to the weight of the whole support vector machine and *w*^−(*p*)^2^^ refers to the weight of support vector machine after feature selection in excluding the *p*th feature. In order to obtain high-quality training data, this paper uses the hybrid network algorithm of the high-order simulated annealing algorithm and *K*-medoid algorithm to mine medical big data.

As shown in Figure 3, the medical big data is mined by using the hybrid network algorithm of the high-order simulated annealing algorithm and *K*-medoid algorithm, and the model of training data set is extracted based on the existing tumor disease medical records. Medical experts should be added to the large medical database to obtain professional experience for a certain kind of disease. Combined with the excellent medical records and prescriptions accumulated by the hospital for a long time, the data are represented by standardized case data and unstructured image data [31–35]. Due to the different medical image manifestations of tumor lesions in different tissues of the human body, it is difficult to collect the clinical characteristics of similar medical records, and the sample size for model training is insufficient. Therefore, this paper selects the small sample classification method, uses training set samples for Feature Engineering, and selects the most effective part of features for model classification under the Spearman method.

### 2.3. Optimization Analysis of Medical Big Data Monitoring Mode

#### 2.3.1. Medical Data Mining Effect Analysis of High-Order Simulated Annealing Combined with *K*-Medoid Algorithm

In order to verify the feasibility of the hybrid neural network with the high-order simulated annealing and *K*-medoid algorithm, the temperature annealing coefficient is set *α* = 0.9, the start stop temperature *t*_*s*_ = 10, the corresponding end temperature *t*_*e*_ is set to 0.01, the inner loop number is set to 100, and the Boltzmann constant *h* is set to 1.

In Figure 4(a), the initial center of cluster 2 is close to the center of cluster. Compared with the more dispersed clusters 0 and 1, the initial center points are in the adjacent boundary range of the objects in each cluster.  Figure 4(b) shows the best clustering effect. For cluster 2, the clustering accuracy reaches 100%. Compared with the scattered cluster 0 and cluster 1, only 4 objects in the two clusters have classification errors; that is, the clustering accuracy is as high as 97.33%. In order to verify the feasibility and efficiency of the proposed high-order simulated annealing combined with the *K*-medoid algorithm hybrid neural network for big data mining, this paper studies the data clustering effect of PAM algorithm, fast *k*-medoids algorithm, *k*-medoids clustering algorithm based on improved granular computing, and the proposed algorithm on iris data set, wine data set, and Pima Indians cubes data set [36, 37].

As shown in Figure 5, on iris data set, the clustering accuracy of the PAM algorithm is 77.56%, that of the fast *k*-medoids algorithm is 89.32%, that of the *k*-medoids clustering algorithm based on improved granular computing is 90.00%, and that of the hybrid neural network of high-order simulated annealing and *K*-medoid algorithm proposed in the study is the highest, 97.33%. On the wine data set, the accuracy of data clustering from high to low is high-order simulated annealing combined with *K*-medoid algorithm, hybrid neural network algorithm, *k*-medoids clustering algorithm based on improved granular computing, fast *k*-medoids algorithm, and PAM algorithm. The corresponding clustering accuracy is 82.11%, 70.79%, 70.79%, and 52.87%, respectively. The clustering algorithm with the highest clustering accuracy on Pima India diabetes data set is the high-order simulated annealing combined with the *K*-medoid algorithm hybrid neural network algorithm proposed in this paper. Its clustering accuracy reaches 70.56%, which is 4.93% higher than that of the *k*-medoids clustering algorithm based on improved granular computing and 8.32% higher than that of the fast *k*-medoids clustering algorithm. Compared with the PAM algorithm, the clustering accuracy is increased by 20.6%. The above results show that the proposed high-order simulated annealing combined with the *K*-medoid hybrid neural network algorithm can effectively mine medical big data.

It can be seen from Table 1 that the fitness of the proposed algorithm is −146.08 and the execution time is 0.750 s on iris, and the two indexes are significantly better than the other two algorithms (fast *k*-medoids algorithm and improved granular *k*-medoids clustering algorithm). On the wine data set, the fitness of the proposed hybrid neural network algorithm is −383, and the execution time is 0.562 a, which is better than the other two algorithms. On Pima India diabetes data set, the fitness of the hybrid neural network algorithm of high-order simulated annealing combined with the *K*-medoid algorithm is –13061701.26 and the execution time is 1.092, which is better than those of the other two algorithms. From the above results, we can know that the proposed big data clustering mining algorithm can complete the data mining and clustering in a shorter time.

## 3. Conclusion

Choosing scientific and effective means to mine the hidden information in medical big data plays an important role in the construction and optimization of cancer disease monitoring mode. Therefore, this paper proposes a clustering algorithm of the high-order simulated annealing neural network algorithm and designs a Spearman + SVM_RFE model to solve the problem of excessive and wrong diagnosis and treatment in the diagnosis and treatment module of tumor disease monitoring mode. The results show that the clustering accuracy of the proposed hybrid neural network algorithm is 97.33%, 82.11%, and 70.56%, the fitness is −146.08, −383.00, and −13061701.26, and the execution time is 0.750 s, 0.562 s, and 1.092 s. It has better clustering accuracy than other clustering methods on the same data set. To sum up, the addition of the high-order simulated annealing neural network algorithm improves the convergence speed of the traditional *K*-medoid algorithm and the clustering accuracy. Model can correctly judge the occurrence of over treatment and wrong treatment in the process of tumor diagnosis and treatment, so as to reduce the incidence of over treatment and wrong treatment, improve the effectiveness of diagnosis and treatment module monitoring, and complete the optimization of tumor disease monitoring mode.

The new algorithm has achieved some results, but it also brings some new problems that need further research. (1) This paper proposes a better method to initialize the *k*-mediods clustering center and improves the *k*-medoids clustering algorithm by using simulated annealing, but it also brings the disadvantages of high time complexity. Therefore, how to reduce the time complexity of the algorithm needs further research. (2) The number of clusters *K* and other parameters in several algorithms proposed in this paper is defined in advance. Whether these parameters can be adjusted adaptively according to the actual algorithm and actual data will be our next research direction. (3) The improved clustering algorithm proposed in this paper only carries out relevant theoretical analysis and relevant experiments in artificial sample object data set and UCI standard data set. Whether it can play a better role in other practical applications needs to be further verified.

## Figures and Tables

**Figure 1:** Flow chart of the simulated annealing algorithm.

**Figure 2:** Tumor disease monitoring mode.

**Figure 3:** Training data extraction process.

**Figure 4:** The results of the algorithm on iris data set.

**Figure 5:** The results of different algorithms on iris data set are compared.

**Table 1:** Comparison of fitness and execution time of different algorithms.

Algorithm	Algorithm fitness comparison			Algorithm execution time comparison(s)		
	Iris	Wine	PId	Iris	Wine	PId
Fast *k*-medoids	−1755.37	−645	−16571303.43	0.809	0.577	1.357
Improved *k*-medoids	−173.88	−431	−14939420.71	1.134	0.655	1.385
The algorithm in this paper	−146.08	−383	−13061701.26	0.75	0.562	1.092

## Data Availability

The data used to support the findings of this study are available from the corresponding author upon request.
